# PPP Financing Model in the Infrastructure Construction of the Park Integrating Artificial Intelligence Technology

**DOI:** 10.1155/2022/6154885

**Published:** 2022-07-14

**Authors:** Xiufeng Wang, Xiaoyan Cui

**Affiliations:** Qingdao Huanghai College, Qingdao 266427, Shandong, China

## Abstract

The objective is to study the application of the Public-Private-Partnership (PPP) financing model in the infrastructure construction of the park. By analyzing the operation model of the PPP financing model, combined with the Artificial Intelligence (AI) technology, the theory mechanism that digital infrastructure construction and Internet use affect the quality of employment is proposed. Based on the selection theory of the PPP model for infrastructure construction projects in industrial parks, the application of the PPP financing model in infrastructure construction of industrial parks is discussed in specific cases. According to the actual situation of the case, the combination of the PPP financing model and government direct investment is proposed, and the predicted income results are given. The results manifest that the total score of the qualitative analysis of the value for money (VFM) of the project of the proposed financing model reaches 85.36 points, greater than 60 points. It indicates that the project has passed the qualitative analysis of VFM, and the profit of the project meets expectations. Among them, the after-tax (AT) internal rate of return of project investment reached 4.3%, and the financial internal rate of return of capital amount reached 4.23% AT, exceeding expectations. It illustrates that the designed PPP financing model meets the requirements. In the infrastructure construction of the park, the combination of digital technology and the PPP financing model can provide a more reasonable financing plan, which is feasible for the infrastructure construction of the park.

## 1. Introduction

As the advanced capital of society, infrastructure construction has the model and function of reshaping economic growth [1–3]. For example, information infrastructure is an important part of maintaining high-quality economic development, and it is the guarantee of advanced technologies such as Artificial Intelligence (AI) and the Industrial Internet. It is a vital part of the government's implementation of macrocontrol in the context of the new era [4–6]. The infrastructure construction of the park is a significant part of the development of the industrial park. However, due to the complex contents of the infrastructure construction of the industrial park, the high project complexity, and the large investment scale of construction projects, a new financing model is urgently needed to solve the dilemma coupled with the problems of later operation and maintenance. The Public-Private-Partnership (PPP) financing model vigorously promoted by China encourages social capital to participate in the investment and operation of various infrastructure projects by means of franchise operations, which is a mechanism of innovation [7–9]. The relationship between the government and social capital is regarded as a partner. They share interests and bear risks together. Government departments can not only effectively use private capital for the construction and operation of projects but also enable private enterprises to obtain open, fair, and access rights. While improving the overall layout of the industrial chain, project operation, and other work efficiencies, it also realizes the adjustment of the entire industry trend. Coupled with the development of advanced computer technologies such as AI, the Internet of Things (IoT), and big data, it can also have different application effects in the infrastructure construction of the park [10–12].

Anwar et al. (2021) [13] pointed out that transportation infrastructure was the backbone of economic development and a major factor in climate change. Therefore, there is a need to transform investments in the transport sector into climate-resilient, low-carbon transport options for sustainable transport infrastructure. For China, such a shift may be necessary from the perspective of a “new urbanization” strategy, and to achieve this strategy, policy adjustments are required. To address this policy-level gap in the literature, the impact of PPP cooperative investment on the transportation sector, renewable energy consumption, and urbanization on China's transportation carbon emissions was explored. Akinsola et al. (2021) [14] studied and assessed the influence of public-private partnerships in energy and financial development on Brazil's ecological footprint, taking into account the role of renewable energy and economic growth using data from 1983 to 2017. The study used several techniques, including the Autoregressive Distributed Lag (ARDL) and Dynamic Ordinary Least Squares (DOLS), to examine the relationship between ecological footprint and determinants while it used a gradual transition causality test to capture causal relationships between sequences in the presence of a single structural break. Abdullah et al. (2020) [15] examined the trust-control relationship in the context of PPP contracts. It draws on the literature and case studies of two UK schools' PPP contracts with varying degrees of trust between partners to illustrate the role of control in building trust in competence and trust in good faith, and how trust in turn affects control. The main reason for the failure of PPP infrastructure projects in conflict areas is insufficient research on PPP risks in these areas and a lack of knowledge to provide effective and feasible solutions to these risks, especially in Afghanistan. Noorzai et al. (2021) [16] conducted research to identify appropriate responses to PPP risks in these projects and to determine priorities for the implementation of risk responses. It suggested that the current PPP financing model is widely used in various industries, but there are few studies on its application in industrial parks.

Using the method of literature research and model implementation, the infrastructure construction mechanism of an AI-based digital smart park is innovatively proposed through the study of the PPP financing model. And for specific industrial park cases, a targeted financing plan combining PPP financing + government direct investment has been established, which can improve the problems existing in the infrastructure construction of industrial parks.

## 2. Materials and Methods

### 2.1. Analysis of the PPP Financing Model

The PPP financing model first originated in the United Kingdom. From the domestic and international current research status, the PPP model is not a unified definition. On account of previous studies, the PPP model is divided into a broad-sense PPP financing model and a narrow-sense PPP financing model [17–19]. In a broad sense, PPP refers to various partnerships between government and private sectors to provide public goods or services. In a narrow sense, it refers to cooperation in the form of a joint investment by the government and the private sector to form a company. In China, the government defines the PPP model as a cooperation model between the government and social capital, which is a long-term cooperative relationship established by government departments and social capital in the field of infrastructure and public services. Social capital is mainly responsible for the design, construction, operation, and subsequent facility maintenance of the project, and its income returns mainly come from “user fees” and “government fees.” The government is responsible for price setting, quality supervision, and other work. The PPP model is actually an institutional innovation, which has a positive impact on the reform and development of the national economy [20–22]. Such a cooperation model can reduce the pressure on the government, improve the efficiency of capital use, and promote the transformation of government functions so that the cooperation between the government and social capital can better serve society and benefit the masses. Besides, it can stimulate the passion and innovation potential of capable people in the society, create more opportunities for enterprises in the normalized economic operation, and pave the way for the development of the mixed-ownership economy. Different types of enterprises can complement each other and learn from each other and reasonably allocate risks and benefits.

There is no single model for the process of project operation. The structure of a representative operation model is displayed in Figure 1.

In Figure 1, the establishment of the PPP model includes 10 steps.

**Step 1 .**

To establish a PPP project.

**Step 2 .**

Obtain debt financing from financial institutions represented by banks.

**Step 3 .**

The PPP financing project obtains the franchise rights.

**Step 4 .**

The contractor and the PPP project company sign a construction contract.

**Step 5 .**

The PPP financing project company pays relevant fees to contractors, suppliers, etc.

**Step 6 .**

The PPP company and the operator sign a contract for later operation and maintenance-related matters.

**Step 7 .**

The PPP financing project company pays the relevant fees to the operator.

**Step 8 .**

The PPP financing company and the insurance company sign an insurance contract.

**Step 9 .**

Source of revenue: user fees, government purchases, etc.

**Step 10 .**

The PPP financing company distributes the corresponding income to the equity capital and debt capital according to the contract.

It denotes that the institutional setting of the PPP model is to allow both parties to participate in the complete project process, and the ultimate goal of the cooperation is to achieve revenue sharing and risk-sharing. It is believed that the PPP model will be intrinsically connected with the current mixed-ownership reform of monopoly industries [23].

### 2.2. Research on Infrastructure Construction of AI-Based Digital Smart Park

The park economy is a significant part and supports the high-quality development of China's economy. Industrial parks in China are quite different in terms of development stage, development level, infrastructure, development scale, and level. The grade and scale, perfection, and carrying capacity of the park's infrastructure construction directly affect the park's comprehensive development capability and business environment. The types of infrastructure in the park are divided into productive infrastructure, productive service facilities, and living infrastructure. Digital infrastructure is an infrastructure system formed by combining a new generation of information technology. The essential characteristics of innovations in Internet technology such as AI and big data play a critical role in economic growth, particularly the commercialization of Internet technology, which further highlights the supporting significance of digital infrastructure to all aspects of social and economic life [24–26]. The theoretical mechanism by which digital infrastructure and Internet use affect employment quality is illustrated in Figure 2:

Figure 2 demonstrates that the application of Internet-based digital technology can effectively reduce the transaction cost of the labor market and can quickly find suitable human capital in the infrastructure construction of the park. The old infrastructure investment model has the disadvantage that the marginal effect is weakened, and it is difficult to provide stamina for the long-term development of the economy. New technology infrastructure is represented by AI, cloud computing, blockchain, etc., as well as computing power infrastructure is represented by the data center and intelligent computing centers, and these new infrastructure models have a huge demand for investment. Meanwhile, it can also completely innovate and upgrade traditional industries and better realize the precise connection between the supply side and the consumer market. It is an investment model that can stimulate both the investment side and the consumer side.

AI often uses deep learning (DL) algorithms in digital infrastructure construction. The database has been established before the DL-related experiments are carried out. Then, a suitable neural network (NN) is selected according to the experimental requirements, and the input data are input into the NN. To make the output data correspond to the target data, the NN will form a set of weight values on each layer of the network. In the process of infrastructure construction of the park, building generative design is an architectural design method based on digital technology, and its mainstream direction is also related to the type of digital technology. In particular, several NN models in DL are commonly used in the generation design method of high-rise residential facades.

The NN consists of three parts, the input layer, the hidden layer, and the output layer. Generative Adversarial Network (GAN) (shown in Figure 3) can be viewed as DL recognizers in the opposite direction. In DL in the field of image recognition, complex data are fed into Deep Neural Networks (DNN) and then gradually compressed. GAN contains two models: a Generative (*G*) and a Discriminative (D), and the two models compete with each other and finally strengthen each other so that the output results are optimal. It can not only identify and classify but also generate and associate. It can achieve different effects when used in high-rise residential facade design in architectural design.

Assuming that *x* represents the real data sample, its distribution obeys the real sample distribution Pdata. *Z* refers to random noise, which obeys the random noise distribution *Pz*. To learn the data distribution through the real data *x* and generate fake data, the random noise vector *z* is input into the generative model to generate fake data denoted as *G*(*z*). The optimization equation of the generative model is as follows:

(1) $$\begin{array}{c} {\text{Max}}_{G}V\left(D,G\right)=E_{z∼pz\left(z\right)}\left[\log\left(D\left(G\left(z\right)\right)\right)\right]. \end{array}$$

After deformation, (2) is obtained as follows:

(2) $$\begin{array}{c} \min_{G}V\left(D,G\right)=E_{z∼pz\left(z\right)}\left[\log\left(1-\left(D\left(G\left(z\right)\right)\right)\right)\right]. \end{array}$$

In the discriminant model *D*, the main responsibility of the discriminator is to determine whether the input data are the real data distribution *x* or the fake data *G*(*z*) generated by the generator. The model outputs a probability value *D*(*x*) by judging whether the input data are true or false, indicating the probability that the input sample is the real data *x*. When the value of the output of the discriminator is closer to 1, the probability that the input sample comes from the real data is higher, and vice versa, which means that the input data have a high probability of coming from the fake data generated by the generator. The objective function of the discriminator is demonstrated as follows:

(3) $$\begin{array}{c} {\text{Max}}_{G}V\left(D,G\right)=E_{x∼p\text{data}\left(x\right)}\left[\log\left(D\left(x\right)\right)\right]+E_{z∼pz\left(z\right)}\left[\log\left(1-D\left(G\left(z\right)\right)\right)\right]. \end{array}$$

The nonlinear activation function is used in DNN to increase the fitting ability of the model. Commonly used activation functions are the Sigmoid activation function, hyperbolic tangent function (Tanh), and Rectified Linear Units (ReLU) function. The expressions are as follows:

(4) $$\begin{array}{c} \text{sigmoid}\left(x\right)=\frac{1}{1+e^{-x}},\\ \tanh\left(x\right)=\frac{e^{x}-e^{-x}}{e^{x}+e^{-x}},\\ \text{relu}\left(x\right)=\max\left(0,x\right). \end{array}$$

The generative design process of high-rise residential facades can be briefly summarized as follows: researchers collect and process data on high-rise residential facades and establish a custom database according to design requirements. The database is used to train the model. The training process of the model is mainly to adjust the parameters. When the generative model can generate better high-rise residential facades, it means that the “generative model” is trained and can be used as a high-rise residential facade generator. At this point, the user draws a schematic diagram that the computer can recognize, and the “generation model” can output design drawings of high-rise residential facades. Generative models using GAN can achieve good results. The schematic diagram of the generation design and implementation process is displayed in Figure 4:

### 2.3. The Application of the PPP Financing Model in the Infrastructure Construction of the Park

In view of the research literature, it is known that the classification of asset returns based on item differentiation theory has been widely used. According to whether the project needs to be charged and whether it can get a return after the operation, it is divided into operating, quasi-operating, and nonoperating projects, and then it is determined whether the project can adopt the PPP financing model, but it will also be flexibly changed with the change of the charging mechanism. The model selection of infrastructure construction projects is illustrated in Table 1:

In Table 1, the final characterization of the project can be evaluated by an expert group, and a score greater than 60 points is considered to have passed the qualitative analysis of the value for money (VFM); otherwise, the strategy will be reestablished. In the cooperation between government and social capital, that is, in PPP projects, the channels for social capital or PPP project companies to obtain investment returns usually include user fees, feasibility gap subsidies, and government payments. For projects that have a clear charging base and operate that can fully cover the investment cost, an appropriate return mechanism should pay for the user. For projects whose operating fees are insufficient to cover investment costs and require government subsidies for some funds or resources, the appropriate return mechanism is the feasibility gap subsidy. For projects that lack a user-payment basis and have no source of operating income, an appropriate return mechanism should be paid by the government. The performance payment shall be paid according to the performance of the PPP project because the infrastructure construction projects of industrial parks usually have a long cycle, high cost, and many participants. There are many risks in the planning and design of the project, the construction and implementation process, and the later operation, so it is necessary to identify and control related risks. The procurement of PPP projects involves many links such as prequalification, bidding, review of bidding documents, and bid winning. The evaluation of bidding documents involves the commercial part (35%), the technical part (35%), and the price (30%).

Taking a large-scale industrial park construction project in Shandong as an example, the PPP model is designed. The infrastructure construction project of the park covers an area of 8.5 km^2^, and most of the surrounding traffic conditions are better in the core area of Transit-Oriented Development (TOD). The total investment amount reaches 15.3 billion yuan, and the cooperation period is 25 years (2019∼2024), including a 60-month construction period and a 20-year operation and maintenance period. The current situation of the project is that if each construction subproject is implemented independently, many border disputes will be formed, which will affect the project process. If it is all managed by the government's direct investment, it is easy to form a situation where the emphasis is placed on construction and less on the operation. If all the PPP models are adopted, one is to use alienated PPP as a financing tool, and illegal borrowing and excessive use of PPP will even exceed 10% of the requirements for the demonstration of financial affordability. Another is to generalize PPP, which does not reflect the problem of “improving the efficiency of the supply of public goods” in PPP, and some projects are not suitable for adopting the PPP model. Therefore, it is comprehensively considered to adopt the government direct investment + PPP model for construction. The schematic diagram of project classification is expressed in Figure 5.

In Figure 5, the government's direct investment part chooses the Engineering-Procurement-Construction (EPC) model of design-procurement-construction integration and the general contractor of the EPC part of the project tenders and the social investors of the PPP part of the project simultaneously. The same winning bidder shall be selected in accordance with the law, and then, the development and construction shall be promoted by the combination model of “EPC + PPP.” The part of EPC that won the bid for this project is also the social capital party of the PPP financing project and can better deal with the construction boundary coordination problem at the same time. EPC construction projects that are required to be suitable for operation and maintenance should still be operated by the PPP project company after the overall construction is completed and enter the operation period. And the construction concept can also be transformed into the long-term “operational performance” of the PPP model. Among them, the AI incubator and its supporting projects include two pieces of land, one of which is comprehensive land for emerging industrial parks. According to the land use index and planning conditions, one of the plots (with a construction area of about 9867.3 m^2^) is used for commercial or business facilities with a service life of 40 years, and the other is a comprehensive land of 2# emerging industrial park (with a construction area of about 36572 m^2^), which is set up according to the nature of the industry and the nature of business offices, and the service life is 50 years.

Combined with the existing financial strength of the area and the planning of the PPP project in the future, the government of this project chooses capital injection and direct investment to support the implementation of the project. Among them, the EPC part adopts the method of direct investment, and the PPP part adopts the method of capital injection. The project is of great significance to the economic development of the area, but the construction investment is large and the financing of funds is relatively difficult. To increase the use efficiency of financial funds, increase the attractiveness of the project, and reduce the payment pressure on government performance during the later operation and maintenance of the project, the government uses direct investment to raise funds for some EPC projects. The PPP project company chooses the project financing method for financing, and only under the premise of obtaining the approval of the government can the expected income rights under the project agreement be set up as pledged security interests for financing or structured financing.

The innovation of setting up the land transfer function in this way is that, on the one hand, it is stipulated that the project company can engage in supporting commercial operations, but in terms of development purposes, the project company is supported to adopt mixed-function uses. When ensuring sufficient commercial supporting construction area in the early stage of the block, the supporting commercial construction area and other construction areas that can be used with public service attributes can be combined and designed. On the other hand, the development and operation of the project by the project company should first meet the needs of the government to attract investment, and the proportion of self-use cannot exceed 15% of the building area. Furthermore, the government, as the capital contributor, that is, one of the project shareholders, has more than one-third of the voting rights and one veto.

When the project is established, VFM evaluation and analysis shall be carried out. For qualitative evaluation, the government organizes a project expert review meeting and invites 7 experts to form a review team. The indicators include the integration degree of the whole life cycle, risk identification and allocation, performance orientation and encouragement of innovation, potential competition degree, capacity of government agency, bankability, project scale, expected service life, major categories of fixed assets, and growth potential value of operating income, a total of 10 projects are numbered ①②③,…,⑩.

## 3. Results and Discussion

### 3.1. Analysis Results of VFM Evaluation of Infrastructure Construction Projects in Industrial Parks

The results of the qualitative evaluation analysis are displayed in Figure 6:

From the comparison in Figure 6, it can be seen that among the basic indicators, the average score of the integration degree of the whole life cycle reaches 89.1 points, which is the highest, and the weight value is 15%. The weight of risk identification and allocation indicators is also 15%, and the average score reaches 79.6 points, which is the lowest. Among the additional indicators, the weight of the project scale and expected service life are both 5%, and the average score is 90.0 points. The lowest score is 85 points for major fixed asset types. Combining all the indicators, the total score of the qualitative analysis of the VFM of the project reaches 85.36 points, and the score is greater than 60 points, indicating that the project has passed the qualitative analysis of VFM, and the PPP model is suitable. In the quantitative evaluation, the results of the calculation and analysis of the risk expenditure within the 25-year cooperation period of the park project are indicated in Figure 7.

Figure 7 refers that in the risk time distribution of the project cooperation period, the single-year risk expenditure in the fifth year of the construction period is the highest, reaching 184.19 million yuan. The total risk expenditure during the construction period is 862.58 million yuan, accounting for about 36.71% of the total project investment. The total risk expenditure during the operation period is 1,487.09 million yuan, accounting for about 63.29% of the total project income. The overall risk expenditure is reasonable. Since the project is a feasibility gap subsidy, most of the financing, construction, operation, and other risks of the projects are transferred to the social capital.

### 3.2. Financial Calculation and Analysis Results

The basic data of project investment are exhibited in Figures 8 and 9.

Figures 8 and 9 indicate that whether it is directly invested by the government or invested by the PPP project company, the amount distribution is relatively reasonable. Construction and installation cost is the largest expense among all costs, and special attention should be paid to the allocation. The financial data of the park project after the calculation are demonstrated in Figure 10:

The income of the PPP project company includes operating income and feasibility gap subsidies. Operating income involves a comprehensive pipe gallery, cultural and sports center, AI incubator, and supporting projects. Figure 10 illustrates that the profit of the project meets expectations. The internal rate of return on project investment after-tax (AT) reaches 4.3%, and the financial internal rate of return on capital amount reaches 4.23% AT, exceeding expectations, indicating that the designed PPP financing model meets the requirements.

Compared with similar PPP financing models (the PPP financing models proposed in [27, 28]), the project follows the work idea of “overall development and overall promotion,” and the implementing agency is the unified owner of the infrastructure construction of the industrial park and adopts the “EPC model + PPP model” for construction. Part of the EPC is directly invested by the government, which is in line with the original intention of the PPP model to “improve the supply efficiency of public goods,” avoids issues such as illegal borrowing and excessive use of the PPP model, and also makes the PPP project within the financial affordability of the local government. In addition, the EPC model is used for the government's independent investment and construction, but the projects with the attributes of operation and maintenance will be handed over to the PPP project company for operation after the completion of the overall construction and the operation period. It also transformed the construction concept of government direct investment in infrastructure projects into the long-term “emphasis on operational performance” of the PPP model and at the same time required the construction unit to ensure the quality of project construction.

## 4. Conclusion

The progress of AI technology has been widely used in various industries. With the rapid expansion of information technology, IoT, 5G, and big data technology, the digital industry and digital economy have become the growth point of the new economy. However, at present, the infrastructure construction of the park faces many problems, especially the financing model. In view of the current situation of financing existing in the infrastructure construction of industrial parks, research is carried out. In the infrastructure construction of AI-based digital smart parks, various NNs of DL are commonly used, especially for GAN, which has advantages in image recognition of architectural design. In view of the financing problem of park construction, a new financing model for infrastructure construction projects is proposed by the PPP financing model. And for the infrastructure construction of a specific industrial park in Shandong, a specific financing plan and a forecast of the operation results of the plan are given. The results signify the effectiveness of the plan and have important theoretical research value. But there are still some deficiencies in the research. In order to improve the operation and maintenance efficiency of the PPP model after the infrastructure of the industrial park is completed, it is an issue that needs further research in the future. Moreover, AI technology covers a wide range, and more case studies are needed to ensure its availability in the construction of industrial parks.

## Figures and Tables

**Figure 1:** Representative operating structure of the PPP model.

**Figure 2:** The theoretical mechanism by which digital infrastructure and Internet use affect employment quality.

**Figure 3:** Structure diagram of GAN.

**Figure 4:** The schematic diagram of the generation design and implementation process.

**Figure 5:** Schematic diagram of park project classification.

**Figure 6:** Qualitative analysis and evaluation results of the VFM of the park project.

**Figure 7:** Calculation results of risk expenditure during the cooperation period.

**Figure 8:** EPC part project.

**Figure 9:** AI incubator and its supporting construction projects.

**Figure 10:** Statistical results of project profitability core indicators.

**Table 1:** PPP model selection for infrastructure construction projects in industrial parks.

Type of project	Types of infrastructure in the park	Financing model
Operational	Water supply and heating facilities, sewage treatment, and publicsupporting property management	PPP model

Quasi-business	Gymnasium, public activity place, and supporting infrastructure	PPP model + government subsidies

Nonoperating	Various demolition projects, municipal road and bridge projects,greening projects, etc.	Government investment

## Data Availability

The data that support the findings of this study are available on request from the corresponding author.
